# Hyperglycemia via activation of thromboxane A2 receptor impairs the integrity and function of blood-brain barrier in microvascular endothelial cells

This article has been retracted.

**DOI:** 10.18632/oncotarget.16273

**Published:** 2017-03-16

**Authors:** Zhihong Zhao, Jue Hu, Xiaoping Gao, Hui Liang, Haiya Yu, Suosi Liu, Zhan Liu

**Affiliations:** ^1^ Department of Neurology, The First Affiliated Hospital (People’s Hospital of Hunan Province), Hunan Normal University, Changsha, Hunan, China; ^2^ Department of Neurology, Changsha Central Hospital, Changsha, Hunan, China; ^3^ Department of Neurology, The People’s Hospital of Xishui, Huangang, Hubei, China; ^4^ Department of Clinical Nutrition and Gastroenterology, The First Affiliated Hospital (People’s Hospital of Hunan Province), Hunan Normal University, Changsha, Hunan, China

**Keywords:** diabetes, thromboxane A2 receptor, blood-brain barrier

## Abstract

Diabetes is one of high risk factors for cardio- and cerebra-vascular diseases, including stroke, atherosclerosis and hypertension. This study was conducted to elucidate whether and how thromboxane receptor (TPr) activation contributes to blood-brain barrier (BBB) dysfunction in diabetes. Human brain microvascular endothelial cells (HBMECs) were cultured. The levels of phosphorylated endothelial nitric oxide synthase (eNOS) at Ser^1177^ (p-eNOS) and Akt at Ser^473^ (p-Akt) were assayed by western blot. Exposure of HBMECs to either high glucose (HG) or thromboxane A_2_ (TxA_2_) mimetic U46619, significantly reduced p-eNOS and p-Akt. These effects were abolished by pharmacological or genetic inhibitors of TPr. HG/U46619-induced suppressions of eNOS and Akt phosphorylation were accompanied by upregulation of PTEN and Ser^380^/Thr^382/383^ PTEN phosphorylation. PTEN-specific siRNA restored Akt-eNOS signaling in the face of TPr activation or HG. The small GTPase, Rho, was also activated by HG stimulation, and pretreatment of HBMECs with Y27632, a Rho-associated kinase (ROCK) inhibitor, rescued HG-impaired Akt-eNOS signaling. In STZ-injected rats, we found that hyperglycemia dramatically increased the levels of PTEN and PTEN-Ser^380^/Thr^382/383^ phosphorylation, reduced both levels of p-eNOS and p-Akt, and disrupted BBB function assayed by Evans blue staining, which were abolished by SQ29548 treatment. We conclude that hyperglycemia activates thromboxane A2 receptor to impair the integrity and function of blood-brain barrier via the ROCK-PTEN-Akt-eNOS pathway.

## INTRODUCTION

Diabetes mellitus is usually associated with the development of cardio- and cerebra-vascular diseases, including stroke, atherosclerosis and hypertension, which is characterized by endothelial dysfunction [1–4]. Prostanoids have critical roles in the development of endothelial dysfunction [5]. Thromboxane A2 (TxA2) perturbs the normal quiescent phenotype of endothelial cells. TxA2 binds to the thromboxane A2 receptor (TPr), activation of which is implicated in atherosclerosis and inflammation [6, 7]. TPr expression and plasma levels of TPr ligands are elevated, both locally and systemically, in several vascular and thrombotic diseases [8]. Importantly, TPr activation induces endothelial cells apoptosis by inhibiting Akt phosphorylation [9]. TPr activation also inhibits vascular endothelial growth factor-induced endothelial cells migration and angiogenesis by decreasing Akt and eNOS phosphorylation [10].

The blood-brain barrier (BBB) protects the brain from potentially neurotoxic substances and facilitates the exchange of nutrients and waste products between the brain and the blood, thus maintaining an optimal extracellular environment for neuronal function [11]. A major role of the blood-brain barrier (BBB) is strict regulation of paracellular permeability. Previous studies showed that the phosphorylation of eNOS at serine 1177 plays an important role in the generation of NO in endothelial cells [12, 13]. Activations of eNOS upstream kinase, such as Akt and AMP-activated protein kinase, increase phosphorylation of eNOS and improve endothelial function [14]. Available data suggest that deficiency of NO mediated endothelial dysfunction in AngII-induced hypertensive mice, as well as in experimental hypercholesterolemia pig [15].

Here, we investigated whether TPr activation promotes BBB dysfunction in diabetes. Our results reveal that activation of TPr abrogates NO production and ROCK-mediated PTEN upregulation is required for TPr-induced BBB dysfunction in diabetes.

## RESULTS

### High glucose and TPr agonist reduce eNOS and Akt phosphorylation in endothelial cells

The important function of endothelial cell is to generate eNOS-derived NO to regulate vascular tone [16]. We firstly investigated the effects of HG on eNOS phosphorylation at Ser1177, which is an eNOS activation site [12]. As shown in Figure 1A, treatment of HMBECs with HG significantly inhibited the phosphorylation of eNOS. As reported previously [13], Akt is an upstream kinase of eNOS. Thus, we examined the effects of HG on Akt activation, as assessed by Ser473 phosphorylation. As expected, we found that both HG reduced the level of Akt phosphorylation at Ser473 (Figure 1B). These data suggest that HG reduces eNOS and Akt phosphorylation in endothelial cells.

**Figure 1:** High glucose and U46619 reduce eNOS-Ser1177 and Akt-Ser473 phosphorylations in HMBECs (**A** and **B**) Confluent HMBECs cultured in 0.5% FBS were pretreated with TPr antagonist (SQ29548, 4 μmol/L) for 20 min and exposed to high glucose (HG, 30 mM) or TPr agonist (U46619, 0.4 μmol/L) overnight. Cells were then harvested for detections of eNOS phosphorylation in A and Akt phosphorylation by western blot in B. (**C**–**E**) HMBECs were pretreated with TPr antagonist (SQ29548, 4 μmol/L) for 20 min and then exposed to high glucose (HG, 30 mM) overnight. Cells were then harvested for detections of AMPK phosphorylation in C, PI3K activity in D, and NO productions in E. *n* = 3, *P < 0.05 *vs*. control, ^#^*P* < 0.05 *vs*. HG or U46619.

To investigate whether HG via TPr activation reduce Akt-eNOS signaling, we tested the effects of TPr agonist U46619 on Akt and eNOS phosphorylations. As indicated in Figure 1A and 1B, treatment of HMBECs with TPr agonist U46619, similar to HG, significantly inhibited the phosphorylations of eNOS and Akt. Co-treatment of TPr antagonist SQ29548 abolished these alternations induced by HG or U46619. Further, SQ29548 did not ablate the reductions of AMPK phosphorylation and PI3K activity induced by HG (Figure 1C and 1D), but reversed NO productions in HG-treated cells (Figure 1E). These data demonstrate that HG possibly inactivates Akt-eNOS signaling in endothelial cells, which is not related to AMPK and PI3K signaling.

### HG via TPr activation inhibits eNOS and Akt phosphorylation in endothelial cells

To further confirm that TPr activation participates in HG-induced inhibition of Akt-eNOS signaling, we transfected HMBECs with TPr-specific siRNA to knockdown TPr. As shown in Figure 2A and 2B, TPr siRNA clearly blocked HG-induced inhibition of eNOS-Ser1177 phosphorylation and Akt-Ser473, while control siRNA did not. These data strongly suggest that TPr activation mediates HG-suppressed Akt-eNOS signaling in endothelial cells.

**Figure 2:** TPr activation is required for HG-induced inhibition of Akt-eNOS signaling in HMBECs. HMBECs were transfected with either control siRNA or TPr siRNA (100 nmol/L) for 48 h and treated with high glucose (HG, 30 mM) overnight Quantitative analysis of (**A**) eNOS phosphorylation and (**B**) Akt phosphorylation in total cell lysates was performed western blot. The blot is a representative of three blots obtained from separated experiments. *n* = 3, *P < 0.05 *vs*. control siRNA alone.

### HG-induced inhibition of Akt-eNOS signaling requires PTEN

To begin to understand what molecules TPr may target to block Akt signaling, we investigated HG-induced changes in PTEN, a lipid phosphatase that participates in Akt dephosphorylation [17]. As shown in Figure 3A, HG induced PTEN phosphorylation at Ser380/Thr382/383, a modification that is essential for PTEN stability. HG also upregulated PTEN protein levels. All these effects induced by HG were blocked by SQ29548.

**Figure 3:** TPr activation meditates HG-impaired Akt-eNOS signaling in a PTEN-dependent manner (**A**) HMBECs were treated with SQ29548 plus high glucose (HG, 30 mM) and harvested for analysis of PTEN-Ser^380^/The^382/383^ phosphorylation and PTEN levels (*n* = 3, *P < 0.05 *vs*. control, ^#^*P* < 0.05 *vs*. HG). (**B**) HMBECs were transfected for 48 h with either control siRNA or PTEN siRNA (100 nmol/L) and treated with HG. Total cell lysates were analyzed by western blot for p-eNOS, eNOS, p-Akt, Akt, and PTEN. (**C**) Quantitative analysis was performed of p-eNOS and p-Akt in B. The blot is a representative of three blots obtained from separated experiments. *P < 0.05 *vs*. control siRNA alone.

To determine whether PTEN is required for HG-induced inhibition of Akt phosphorylation, we transfected HMBECs with PTEN-specific siRNA. Transfection of PTEN siRNA, but not control siRNA, markedly reduced endogenous PTEN in HMBECs (Figure 3B). However, PTEN-specific siRNA did not alter Akt-Ser473 or eNOS-Ser1177 phosphorylation. Importantly, HG-induced inhibition of Akt and eNOS phosphorylation was blocked by transfection of PTEN-specific siRNA, but not control siRNA (Figure 3C). Taken together, these results imply that HG-induced impairment of endothelial Akt signaling requires PTEN.

### HG via TPr activation disrupts BBB integrity

We then determined the effect of HG on the paracellular permeability in cultured HBMEC monolayer on transwell filters. As depicted in Figure 4A, HG significantly increased the leakage of FITC-dextran of 150 kDa after 24-hour incubation. Conversely, 24-hour incubation of HBMEC with HG reduced *trans*-endothelial electrical resistance across a monolayer (Figure 4B), accompanied with decreased protein expressions of tight-junction proteins, occludin and claudin-5 (Figure 4C).

**Figure 4:** Antagonist of TPr by SQ29548 improves tight-junction in HBMECs incubated with HG. HMBECs were treated with SQ29548 plus high glucose (HG, 30 mM) for 24 hours (**A**) Confluent monolayer of HBMECs was cultured on Transwell filters and the diffusion of FITC-conjugated dextran (150 kDa; 100 μg/ml) was measured. (**B**) *Trans*-endothelial electrical resistance was measured in confluent monolayer of HBMECs. (**C**) Representative Western blot of tight-junction proteins (occludin and claudin-5). Control was set up as 100%. Data are expressed as the mean ± SEM. N is 5 in each group. *P < 0.05 *VS* control group. NS indicates no significance. (**D**)The morphology of tight-junction was determined by using staining F-actin.

To determine the role of TPr in HG-induced disruption of BBB, HBMECs were pretreated with SQ29548 followed by HG incubation. As shown in Figure 4A–4D, antagonist of TPr by SQ29548 abolished these abnormalities including increased the leakage of FITC-dextran, reduced *trans*-endothelial electrical resistance across a monolayer, decreased protein expressions of tight-junction proteins, occludin and claudin-5, and disrupted morphology of tight junction. These data suggest that TPr activation contributes to BBB dysfunction induced by HG.

### Rho/ROCK participates in HG-reduced Akt-eNOS signaling

In human ECs, Rho/ROCK negatively regulates eNOS phosphorylation by inhibiting Akt [18]. However, whether the Rho kinase pathway participates in HG-induced inhibition of Akt-eNOS signaling is unknown. To investigate whether Rho participates in TxA2 signaling, we determine if stimulation of HG activates Rho. Rhotekin pull-down assays revealed that HG did stimulate Rho activation (Figure 5A), consistent with the ability of TPr agonist to activate Rho in prostate carcinoma PC-3 cells [19]. This activation was attenuated by pretreatment of cells with SQ29548, suggesting that HG activates Rho through TxA2 receptor stimulation.

**Figure 5:** Rho/ROCK participates in HG-induced inhibition of Akt-eNOS signaling (**A**) HMBECs were treated with SQ29548 plus high glucose (HG, 30 mM) for 24 hours. Active Rho (GTP bound) in total cell lysates was analyzed by using Rhotekin pull-down assays. (**B** and **C**) HMBECs were treated with Y27632 (10 μM) plus high glucose (HG, 30 mM) for 24 hours. Western blot analysis of p-Akt and p-eNOS in B, and p-PTEN and PTEN in C was performed. The blot is representative of three blots obtained from three independent experiments. *P < 0.05 *vs*. control, ^#^*P* < 0.05 *vs*. HG.

To investigate the requirement for Rho/Rho-associated kinase (ROCK) in HG-induced inhibition of Akt-eNOS signaling, we evaluated the effects of Y27632, a specific inhibitor of ROCK [20]. As shown in Figure 5B, Y27632 pretreatment blocked HG-induced inhibition of Akt and eNOS phosphorylation in HMBECs. Y27632 also considerably disrupted HG-induced increases in PTEN and p-PTEN (Figure 5C). Taken together, these data show that Rho activation is required for HG-induced inhibition of Akt and eNOS signaling.

### Antagonist of TPr by SQ29548 attenuates hyperglycemia-induced dysfunction blood-brain barrier in rats

At last we determined whether antagonist of TPr improved BBB function in diabetic rats. To test this notion, mice were injected rats with STZ to induce hyperglycemia. Permeability of the BBB was assessed using EB, a dye that tightly binds to albumin as described previously [21]. SQ29548 had no effects on blood glucose in mice injected with or without STZ (Data not shown). Under normal physiological circumstances, albumin is prevented from entering the brain neutrophil by the BBB. Thus, the amount of EB dye within the brain tissue can be used to quantify BBB disruption. During hyperglycemia, a significant increase in BBB permeability occurred compared to saline (Figure 6A and 6B). Treatment with TPr antagonist SQ29548 resulted in a marked reduction in BBB permeability. Simultaneously, SQ29548 significantly increased both levels of occludin and claudin-5 (Figure 6C). All data support that TPr inactivation improved BBB function in diabetes.

**Figure 6:** Antagonist of TPr by SQ29548 attenuates hyperglycemia-impaired integrity and function of blood-brain barrier in rats Male rats received STZ injection (50 mg/kg/day) for 5 consecutive days and then treated with or without SQ29548. At the end of experiment, rats were sacrificed under euthanasia to detect BBB permeability. (**A**) Representative images of whole brains stained by Evans blue dye. (**B**) Evans blue extravasations in brains. (**C**) Protein expressions of occludin and claudin-5 by Western blot. Data are expressed as the mean ± SEM. Five mice were in each group. *P < 0.05 *VS* control. ^#^*P <* 0.05 *VS* STZ alone.

### TPr activation mediates hyperglycemia-reduced Akt-eNOS signaling in rats

We finally determined the effects of hyperglycemia on p-Akt and p-eNOS *in vivo*. As shown in Figure 7A–7C, aortic levels of eNOS and Akt phosphorylations were significantly decreases in diabetic rats. Differently, the levels of PTEN and p-PTEN were reduced by hyperglycemia. Importantly, inhibition of TPr by SQ29548 abolished these abnormalities induced by hyperglycemia in rats. Overall, these results suggest that TPr activation mediates hyperglycemia-reduced Akt-eNOS signaling *in vivo*.

**Figure 7:** TPr activation mediates hyperglycemia-reduced Akt-eNOS signaling in rat brains (**A**–**C**) Brain homogenates from STZ-injected diabetic rats administrated with vehicle or SQ29548 were analyzed for the levels of total and phosphorylated (A) eNOS (phosphorylation at Ser^1177^), (B) Akt (phosphorylation at Ser^473^), and (C) PTEN (phosphorylation at Ser^380^/Thr^382/383^). All data were expressed as mean ± SEM. N is 10–15 in each group. *P < 0.05 vs. Vehicle group. ^#^*P <* 0.05 vs. Diabetes. (**D**) Proposed pathway underlying hyperglycemia-induced BBB dysfunction.

## DISCUSSION

In the present study, we have for the first time provided evidences that hyperglycemia via TPr activation induces BBB dysfunction *in vitro* and *in vivo*. Furthermore, we have characterized that activation of TPr by HG stimulates PTEN to suppress Akt-eNOS signaling, resulting in brain arterial endothelial cells (Figure 7D). These findings support a key role of TPr activation in the formation of stroke in diabetes.

These data may have important implications in clinical settings. TPr activation is thought to contribute to the development of hypertension because diabetic mice have elevated PTEN levels. Our results have uncovered a novel mechanism whereby TPr activation induces impairments in endothelial Akt-eNOS signaling, which may cause increased permeability of brain vascular endothelium layer, contributing to stroke. We previously have reported that AMPK activation maintains endothelial tight junctions in brain microvascular of BBB upon long-term exposure to LPS [22, 23]. Although we did not examine the role of AMPK-signaling in diabetic BBB dysfunction, this study indicated that inactivation of PTEN-Akt-eNOS signaling by hyperglycemia via TPr activation contributes to BBB dysfunction. Importantly, agonist of TPr by SQ29548 reversed hyperglycemia-induced BBB disruption in diabetic rats, indicating that TPr activation may help account for the detrimental effects of hyperglycemia on cerebrovascular complications.

A limitation of this study is that we used STZ-induced diabetes in rat as a risk factor to induce endothelial dysfunction. STZ is known to destroy islets of Langerhans in the pancreas [24], therefore, the induced persistent hyperglycemia in the animals resembles insulin-dependent type 1 diabetes in humans. The major cardiovascular complications of diabetes, including hypertension, atherosclerosis, and stroke, are characteristic for type 2 diabetes or insulin resistance [25]. A better model is obesity db/db mice, which is quite similar to type 2 diabetes [26], rather than STZ-induced diabetic model. Whether endothelial dysfunction in obesity db/db mice is mediated by TPr activation need our further investigations.

## MATERIALS AND METHODS

### Materials

Primary antibodies against PTEN, phospho-PTEN-Ser^380^/Thr^382/383^, Akt, phospho-Akt-Ser^473^, eNOS, phospho-eNOS-Ser^1177^, and β-tubulin were obtained from Cell Signaling Technology (Beverly, MA). All siRNAs were from Santa Cruz Biotechnology Inc. (Santa Cruz, CA). The siRNA delivery agent, Lipofectamine 2000, was from Invitrogen (Carlsbad, CA). Streptozotocin (STZ), U46619, SQ29548, and rabbit polyclonal antibodies against TPr were purchased from Cayman Chemical (Ann Arbor, MI). All other chemicals and organic solvents were of the highest grade and were obtained from Sigma-Aldrich (St Louis, MO).

### Cell culture and transfection of siRNA into cells

Human brain microvascular endothelial cells (HBMECs) purchased from Invitrogen, Gibco Cell Culture (Portland, OR) were cultured as described previously [27]. Transient transfection of siRNA was carried out according to Santa Cruz’s protocol as described previously [28].

### Western blot analysis

As described previously [29], cell lysate containing 20–50 μg of protein were separated on a polyacrylamide gel with Tris-glycine-SDS and transferred onto nitrocellulose membranes for 2 h. After incubation of membrane with primary antibody and secondary antibody, reactive bands were detected using ECLTM Western Blotting Detection Reagents (Amersham).

### Rhotekin pull-down assay for RhoA activation

HBMECs were plated in 0.5% serum medium in 10-cm culture dishes. After treatment, cells were rapidly lysed on ice and processed for assay of the levels of GTP-bound RhoA. Assays were performed according to the manufacturer’s instructions (Cell biolabs, Inc) as described previously [30].

### Permeability of the BBB *in vitro*

HBMECs were cultured on Costar Transwell filters (pore size 0.4 μm; Corning, NY, USA) that were coated on the upper side with fibronectin (Sigma–Aldrich) in endothelial cell growth medium mixed with astrocyte-conditioned medium at a 1:1 ratio as described previously [22].

### Determination of trans-endothelial electrical resistance

Determination of *trans*-endothelial electrical resistance across the monolayer of HBMECs was measured using the Millicell-ERS (Millipore) as described previously [22].

### Induction of hyperglycemia and animals experimental protocol

Male Sprague-Dawley (SD) rats (8 ± 2 weeks old, 180 ± 20 g) were purchased from Hua-Fu-Kang Animal Company (Beijing, China). A low-dose (50 mg/kg/day for 5 consecutive days) STZ induction regimen was used to induce pancreatic islet cell destruction and persistent hyperglycemia as described previously [31]. This study was carried out in strict accordance with the recommendations in the Guide for the Care and Use of Laboratory Animals of the National Institutes of Health. The protocol was approved by the Committee on the Ethics of Animal Experiments of Hunan Normal University.

### Evaluation of BBB permeability *in vivo*

As described previously [32], rats were injected intraperitoneally with 1 ml of 1% Evans Blue dye and perfused with PBS to remove intravascular Evans Blue dye under anesthesia. Then, the whole brain was weighed, homogenized, and the Evans blue dye was extracted. The extracted supernatant was measured by absorbance spectroscopy at 620 nm for Evans blue determination. Calculations were based on external standards in the same solvent.

### Statistical analysis

Values are expressed as mean ± SEM. Statistical comparisons of vasodilation were performed using ANOVA. Intergroup differences were analyzed using Bonferroni’s post-test. Analysis of time-course studies was performed with repeated measures ANOVA. *P* values less than 0.05 were considered as significant.
